RETRACTED

# Application Value of Health Education Combined with Aerobic Exercise in Nursing of Patients with Mastitis Found in Physical Examination

**DOI:** 10.1155/2022/8369626

**Published:** 2022-03-29

**Authors:** Xiuxia Wang, Xianglian Sun

**Affiliations:** ^1^Health Management Center, Qingdao Jiaozhou Central Hospital, Qingdao 266300, Shandong, China; ^2^Thyroid and Breast Surgery Area I, Weifang People's Hospital, Weifang 261041, Shandong, China

## Abstract

**Objective:**

To explore the application value of health education combined with aerobic exercise in patients with mastitis found in physical examination.

**Methods:**

The clinical data of 100 patients with mastitis who underwent physical examination in the physical examination center of our hospital from October 2020 to October 2021 were retrospectively analyzed. According to the order of physical examination, they were equally split into experimental group and control group. The control group received the routine clinical intervention, while the experimental group received health education combined with aerobic exercise to evaluate the clinical effects of different intervention modes on patients with mastitis.

**Results:**

Compared with the control group, the experimental group after intervention achieved notably higher scores of CD-RISC, self-management ability, and mastitis-related knowledge (*P* < 0.001), lower scores of breast pain, skin color, and local mass diameter (*P* < 0.001), and a higher SF-36 score (*P* < 0.001).

**Conclusion:**

The clinical intervention combining health education with aerobic exercise in patients with mastitis found in the physical examination is an effective method to improve their mood state and self-management ability, and further research will help provide a good solution for such patients.

## 1. Introduction

Mastitis is an inflammation of the breast caused by the infection that carries a risk in women of any age but is most common in lactating women [1]. The clinical manifestations such as swelling, pain, and redness of breast tissues and local breast mass damage can also lead to pyogenic infection, triggering chills, and fever all over the body in patients [2, 3]. In recent years, the prevalence of nonlactating mastitis has increased year by year, which has a serious impact on the quality of life of patients due to the complex clinical manifestations and difficulty in its treatment. Since mastitis can be found through physical examination, clinical intervention for patients with mastitis found in the physical examination is the key to improving symptoms and enhancing the quality of life [4, 5]. In addition to the necessary drug treatment, scientific rehabilitation exercise and health education are also effective measures to improve the outcomes of mastitis [6]. Health education is conducive to deepening patients' understanding of their own diseases, enhancing their self-care ability, improving treatment compliance, and establishing healthy living habits, which has been confirmed in diseases such as vitiligo, adolescent idiopathic scoliosis, and osteoporotic vertebral compression fractures [7–9]. Aerobic exercise, a comprehensive exercise, can not only relieve the physical and mental health of patients but also coordinate muscle contraction and exercise ability. The implementation of aerobic exercise can adjust the respiration of patients, improve physiological metabolism, promote the growth of bone mineral density, and facilitate the recovery of the body [10]. In addition, regular aerobic exercise can also stimulate the secretion of dopamine and divert the attention of patients, thus eliminating adverse emotions [11]. At present, no research has confirmed the application value of health education combined with aerobic exercise in patients with mastitis found in physical examination. In view of this research vacancy, this study carried out a combined clinical intervention on the subjects to provide more clinical evidence-based proof for such patients.

RETRACTED

## 2. Materials and Methods

### 2.1. General Data

The subjects were 100 patients diagnosed with mastitis who underwent physical examination in the physical examination center of our hospital from October 2020 to October 2021. According to the order of physical examination, they were equally split into experimental group and control group. This study conformed to the Declaration of Helsinki [12].

### 2.2. Inclusion and Exclusion Criteria

Inclusion criteria: (1) patients met the diagnostic criteria for mastitis, such as the hard masses with unclear boundary and poor activity, accompanied by symptoms such as redness, swelling, heat and pain, local pain of breast, and galactapostema; (2) B-ultrasonography showed irregular low-echo masses, with a few liquid echo areas occasionally; and (3) patients aged 18–60 years old and their families were familiar with the precautions of aerobic exercise.

Exclusion criteria: (1) patients with organic mental disorder and mental illness; (2) patients with regular exercise habits before enrollment; and (3) patients with serious underlying diseases, such as diseases in brain, heart, liver and kidney, and hematopoietic diseases.

### 2.3. Methods

The control group was given routine clinical intervention after diagnosis. The medical and nursing staff helped patients complete relevant examinations (including physical examination, routine blood test, and breast ultrasonography) and various nursing operations, eliminated their tension and fear, and ensured that they could cooperate with doctors in treatment. Any abnormalities in patients were timely reported to competent doctors. The patients were guided to face life optimistically and establish confidence in treatment [13, 14].

RETRACTED

The experimental group received health education combined with aerobic exercise. Health education was implemented as below. Differentiated intervention strategies and education contents were provided by the nursing staff according to the education levels, comprehension, occupation, and social status of each patient. The etiology, pathogenesis, and other in-depth medical knowledge of mastitis were illustrated to patients with a high education level, while simple and plain words were applied to those with a low education level. At the same time, patients with mastitis were instructed to master a healthy lifestyle and develop good hygienic habits. During intervention, four health lectures on disease knowledge were conducted to improve the self-management ability of patients, including healthy lifestyle, healthy exercise behaviors, correct medication, and healthy dietary behaviors.

Aerobic exercise was carried out as below. According to the individual characteristics of patients, the rehabilitation physicians formulated corresponding exercise strategies. The patients carried out 2-3 times of exercise each week in the first three weeks, with the exercise time at 15–20 min each time and no intense exercise and then gradually increased the time. In the 10th week, the exercise time was increased to 35–40 min and the exercise intensity was assessed based on the patients' heart rates. Maximum heart rate = 220 − patient age. Exercise intensity was 50% of the highest heart rate in the 1–6 weeks, 60% of that in the 7–10 weeks, and 70% of that after the 10th week. The patients were guided to correctly calculate their heart rates and control the rates during exercise. Aerobic exercise included warm-up exercise, real exercise, and relaxation at a ratio of 1 : 3 : 1 in time. Various sports were chosen according to personal preferences and objective needs, such as yoga, jogging, swimming, and walking. Medical staff grouped patients according to their living areas, same interests and hobbies, and similar ages and encouraged them to engage in the same exercise and communicate with each other. At the same time, regular health education was carried out to inform patients of the benefits of adhering to aerobic exercise for the treatment of mastitis, the choice of exercise methods, and self-rescue and treatment for abnormalities in exercise. Patients were regularly followed up to ask about their exercise and physical status. The aerobic exercise was carried out for 10 weeks.

RETRACTED

### 2.4. Observation Indicators

The resilience scale (CD-RISC) [15] was adopted for evaluating the psychological state of patients, which was composed of three factors (resilience, confidence, and optimism) and 25 problems in total. The 5-level scoring method (0–4 points) was used for each problem, and a higher score demonstrated a better psychological state.

In terms of local situation of the affected breast, 0 point was for no local pain, 2 for mild and tolerable pain, 4 for obvious pain that did not affect sleep, and a score of 6 points was for severe local pain that seriously affected work and sleep. As for local skin condition, 0 point was for normal local skin color with no heat sensation, 2 for normal local skin color with slight heat sensation, 4 for red local skin with burning sensation, and 6 for local skin ulceration. Concerning local mass diameter, 0 point was for no local mass, 2 for a local mass diameter ≤2 cm, 4 for a local mass diameter of 2–4 cm, and 6 for a local mass diameter >4 cm.

The self-management ability of patients was evaluated according to the self-designed questionnaire on self-management ability of patients with mastitis in our hospital. The questionnaire included daily life management, abnormal handling, exercise management, and self-management confidence. Each item contained five questions, and each question had five grades of positive scores (1–5 points). A higher score represented better self-management ability of the subjects.

The self-made questionnaire on disease knowledge of mastitis in our hospital was used to evaluate the mastery of disease knowledge of both groups, including the pathogenesis of mastitis, treatment methods, daily nursing methods and principles, and regular return visits. The full score was 100 points, and a score ≥80 points was regarded as qualified for the mastery of mastitis-related knowledge.

The MOS 36-item short-form health survey (SF-36) [16] was used to evaluate the quality of life of both groups after intervention, including somesthetic sensation, health perception, sleep quality, and social integration, with each item scoring 25 points, and a total score of 100 points. A higher score indicated better quality of life.

### 2.5. Statistical Methods

The data were processed by the professional statistical software SPSS26.0 and graphed by GraphPad Prism 7 (GraphPad Software, San Diego, USA). The enumeration data were tested by *X*^2^ and expressed as (*n* (%)), while the measurement data were tested by the *t* test and expressed as mean ± SD. When *P* < 0.05, the differences were statistically significant.

RETRACTED

## 3. Results

### 3.1. General Information

No notable differences in the average age, breast feeding history, residence, family income, and other general information were observed between the two groups (*P* > 0.05), see Table 1.

### 3.2. CD-RISC Scores

Figure 1 demonstrated a notably higher CD-RISC score in the experimental group after intervention than in the control group (*P* < 0.001).

### 3.3. Local Situation of the Affected Breast

After intervention, the scores of breast pain, skin color, and local mass diameter in the experimental group were obviously lower than those of the control group (*P* < 0.001), see Table 2.

### 3.4. Self-Management Ability

The scores of self-management ability after intervention were notably higher in the experimental group than in the control group (*P* < 0.001), as presented in Table 3.

### 3.5. Scores of Mastitis-Related Knowledge

The score of mastitis-related knowledge was higher in the experimental group than in the control group (*P* < 0.001), see Figure 2.

### 3.6. Quality of Life

After intervention, the SF-36 score was higher in the experimental group than in the control group (*P* < 0.001), see Figure 3.

## 4. Discussion

Characterized by repeated attacks and difficult recovery for metastasis, mastitis seriously affects patients' physical and mental health, with no specific and effective treatment in modern medicine [17]. Surgery can lead to breast deformation, seriously affecting appearance and causing a great psychological impact on patients. Some scholars [18] have suggested that the implementation of effective clinical interventions can largely reduce the clinical symptoms of mastitis and enhance the quality of life of patients with the administration of conventional western medicine. With the rapid replacement of clinical nursing modes, diversified nursing forms are favored by the majority of patients. As health education is applied in more diseases with the core of changing patients' behavioral habits, its nature, purpose, and tasks must be closely integrated with science [19]. The ultimate goal of health education is to change people's behaviors. Health education for patients with mastitis, a chronic disease characterized by difficult recovery for metastasis, can significantly improve their daily living habits, help them establish a good lifestyle, and improve their prognosis.

Aerobic exercise, including the common forms of swimming, walking, skating, riding a bike, and rhythmic exercise, has always been a healthy exercise modality advocated by medical workers, already with several studies on it [20]. This exercise mode can accelerate the blood circulation of the human body, promote the metabolism of the tissues, improve body function, and provide sufficient protection for the operation of other systems in the body, which has been confirmed in diseases such as chronic obstructive pulmonary disease, senile cognitive impairment, and nonalcoholic fatty liver disease [21]. Based on the previous clinical experience, this study aimed to bring an evidence-based basis for patients with mastitis through the implementation of aerobic exercise combined with health education. The CD-RISC score was higher in the experimental group than in the control group after intervention (*P* < 0.001). Clinical studies [22] found that after conducting health education to hospitalized patients with type 2 diabetes, their emotions were obviously improved compared with before the intervention, which once again confirmed the conclusion of this study. Due to patients' lack of awareness of their own diseases and stronger physical pain caused by the disease, the patients are prone to adverse emotions with an increased psychological burden resulting from the economic pressure. In this study, health education was carried out to enhance the awareness of patients with mastitis, which eliminated their fear and tension to a large extent and boosted their confidence in treatment. In aerobic exercise, the nervous system releases weak electrical stimulation that effectively relieves muscle tension and mental depression, relaxes the cerebral cortex, and alleviates psychological tension [23, 24]. The score of mastitis-related knowledge was higher in the experimental group than in the control group (*P* < 0.001), suggesting that the combined intervention greatly increases the patients' awareness of their own disease, improves their tolerance to relevant medical operations, enables them to actively cooperate with the diagnosis and treatment, and enhances their confidence in treatment. A previous study [25, 26] has found that patients may lack entertainment, communication, and cooperation during exercise if aerobic exercise is carried out in an individual form, resulting in low exercise compliance. Therefore, in this study, medical staff grouped patients according to their living areas, same interests and hobbies, and similar ages, and those in the same group could jointly engage in the same exercise and communicate with each other, thus enhancing exercise compliance. A study [27–29] has shown that aerobic exercise with appropriate intensity can maintain normal cytokine levels, in which the patients can fully communicate with the surrounding patients and friends while exercising, thereby relieving their emotions.

RETRACTED

Due to limited research conditions, this study has a short follow-up time and lacks research on the recurrence of disease after intervention. Therefore, the experimental design will be improved in the subsequent studies to provide more evidence-based proof for the clinical intervention of mastitis.

## Figures and Tables

**Figure 1:** Comparison of CD-RISC scores after intervention (mean ± SD). Note: the abscissa was the experimental and control groups, and the ordinate was the CD-RISC score (points). The CD-RISC scores of the experimental and control groups were 63.70 ± 5.89 and 58.72 ± 3.36, respectively. ^*∗*^A notable difference in the CD-RISC scores between the two groups (*t* = 5.193, *P* < 0.001).

**Figure 2:** Comparison of scores of mastitis-related knowledge after intervention (mean ± SD). Note: the abscissa was the experimental and control groups, and the ordinate was the score of mastitis-related knowledge (points). The scores of mastitis-related knowledge in the experimental and control groups were 78.42 ± 5.88 and 63.08 ± 6.16), respectively. ^*∗*^A notable difference in the scores of mastitis-related knowledge between the two groups (*t* = 12.737, *P* < 0.001).

**Figure 3:** Comparison of SF-36 scores (mean ± SD). Note: the abscissa was the experimental and control groups, and the ordinate was SF-36 score (points). The SF-36 scores of the experimental and control groups were 76.26 ± 6.37 and 71.22 ± 2.25, respectively. ^*∗*^A notable difference in the SF-36 scores between the two groups (*t* = 5.275, *P* < 0.001).

**Table 1:** Comparison of general data.

Items	Experimental group	Control group	*X* ^2^/*t*	*P*
Average age (mean ± SD, yrs)	44.52 ± 12.64	44.84 ± 10.87	0.136	0.892
BMI (mean ± SD, kg/m^2^)	21.72 ± 0.91	21.75 ± 1.02	0.155	0.877
Breast feeding history				
Yes	29 (58.00)	32 (64.00)	0.378	0.539
No	21 (42.00)	18 (36.00)		
Nipple inversion				
Yes	34 (68.00)	35 (70.00)	0.047	0.829
No	16 (32.00)	15 (30.00)		
Family income				
≥3000 yuan/(month person)	27 (54.00)	29 (58.00)	0.162	0.687
<3000 yuan/(month person)	23 (46.00)	21 (42.00)		
Residence (*n* (%))				
Urban area	27 (54.00)	31 (62.00)	0.657	0.418
Rural area	23 (46.00)	19 (38.00)		
Education (*n* (%))				
College degree and above	7 (14.00)	9 (18.00)	0.298	0.585
Senior high school	12 (24.00)	13 (26.00)	0.053	0.817
Junior high and below	31 (62.00)	28 (56.00)	0.372	0.542

**Table 2:** Local situation of the affected breast (mean ± SD, points).

Group	*n*	Breast pain	Skin color	Local mass diameter
Experimental group	50	1.36 ± 1.24	1.64 ± 1.50	1.92 ± 1.45
Control group	50	3.52 ± 1.37	3.72 ± 1.57	3.96 ± 1.78
*t*		8.266	6.773	6.283
*P*		<0.001	<0.001	<0.001

**Table 3:** Comparison of self-management ability after intervention (mean ± SD, points).

Group	*n*	Daily life management	Abnormal handling	Exercise management	Self-management confidence
Experimental group	50	20.60 ± 2.36	19.34 ± 2.33	19.16 ± 2.77	21.30 ± 2.12
Control group	50	16.08 ± 2.18	16.48 ± 2.48	16.06 ± 2.04	14.98 ± 1.92
*t*		9.948	5.943	6.372	15.624
*P*		<0.001	<0.001	<0.001	<0.001

RETRACTED

## Data Availability

The data used to support the findings of this study are available on reasonable request from the corresponding author.
